The article "Untargeted Metabolite Profiling of Specialty Rice Grains Using Gas Chromatography Mass Spectrometry" was published in 2022. Journal: Int J Anal Chem.

# Untargeted Metabolite Profiling of Specialty Rice Grains Using Gas Chromatography Mass Spectrometry

**DOI:** 10.1155/2022/2558072

**Published:** 2022-09-19

**Authors:** Rohit Kambale, M. Raveendran, J. Ramalingam

**Affiliations:** Department of Plant Biotechnology, Tamil Nadu Agricultural University, Coimbatore, Tamil Nadu, India

## Abstract

With-ever increasing demand food grains for the increasing population, it has also increased the importance of quality rice with nutritional and therapeutic properties. The quality of rice includes nutritional value, therapeutic properties, and further generation of aroma. Initial studies on sensory analysis using potassium hydroxide (1.7% KOH) identified the presence of a distinct aroma of the traditional rice cultivar Chakhao Amubi in comparison with other aromatic rice varieties were conducted. The metabolomic profiling of aromatic rice grains Chakhao Amubi, Pusa Basmati 1, and nonaromatic rice, Improved White Ponni was attempted to use gas chromatography-mass spectrometry (GC-MS). A total of fifty volatile aromatic compounds, including aromatic hydrocarbons, alkanes, alkenes, ketones, and aromatic aldehydes, have been identified. Detected compounds include six crucial volatile i.e., pentanal, hexanal, 2-pentylfuran, pyridine, (Z)-7-Decenal, and Mesitylene for distinct flavor and presence of aroma in Chakhao Amubi. The findings showed a distinct difference in the metabolic profile of Chakhao Amubi compared to Pusa Basmati 1 and Improved White Ponni. Thus, this study paved the way for a new understanding of the aromatic aspects of traditional rice germplasm and its utilization in rice breeding programs to improve the aroma, therapeutic, and nutritional characteristics of rice.

## 1. Introduction

Being a staple food for more than half of the world's population, rice holds a key position in achieving food security. It is predicted that the global population will reach beyond 9.7 billion in 2050, which necessitates a doubling of rice production to ensure food and nutritional security [1]. Even though rice serves as a staple food for the majority of the population, its consumer preference varies greatly between different countries. In India, preference for rice quality (size, taste, and aroma) differs between regions [2]. Next to the grain size and cooking quality, aromatic rice is highly preferred by the majority of consumers because of the fragrance and its unique taste. Aromatic rice is considered to be the most precious asset of rice diversity to India and fetches a premium price (3 times higher price than nonaromatic rice) in the export market. Among the various fragrant rice cultivars, Sadri (Iran), Basmati (India and Pakistan), Jasmine (*indica* rice from Thailand) and a few tropical *japonicas* are ruling the market [3]. Systematic screening of >250 volatile and nonvolatile compounds in aromatic and nonaromatic rice varieties identified a compound, 2-acetyl-pyrroline (2AP), majorly responsible for the production of pop-corn like aroma in rice [4, 5]. Aromatic rice varieties greatly differ in their 2AP content, as reported in Basmati (0.34 ppm), Jasmine (0.81 ppm), and Texmati (0.53 ppm). Later, it was found that 2AP has present in both aromatic and nonaromatic rice varieties, but they differed in concentration [6]. In addition to 2-acetyl-1-pyrroline, other novel compounds like 2-amino acetophenone and 3-hydroxy- 4, 5-dimethyl-2 (5H) -furanone in Basmati 370 [7] and guaiacol and indole and p-xylene in Black rice [8] were also reported to contribute for a unique flavor in the rice. In addition to 2-acetyl-1-pyrroline, more than 100 volatile organic compounds, namely, hexanal, nonanal, octanal, nonenal, (E, E)-2, 4-nonadienal, heptanal, (E)-2-octenal, 4-vinyl phenol, 4-vinyl guaiacol, 1-octen-3-ol, decanal, have been reported. [9, 10].

The article "Untargeted Metabolite Profiling of Specialty Rice Grains Using Gas Chromatography Mass Spectrometry" was published in 2022. Journal: Int J Anal Chem.

Recent advancements in molecular genetics and sequencing enabled the molecular dissection of aroma in rice. QTL mapping and comparative sequence analysis of OsBADH2 gene on chromosome 8 between the aromatic rice KDML105 and a nonaromatic rice Nipponbare identified key mutations in the exon 7 of OsBADH2 namely, two base pair substitutions, one at 730 bp (A to T), another base pair substitution at 732  bp (T to A), and an 8-bp deletion “GATTAGGC” starting from 734  bp [11]. Similar studies in the aromatic rice variety Kayeema also identified an 8  bp deletion in the exon 7 of OsBADH2 [12, 13]. In addition to the fragrance gene OsBADH2 on chromosome 8, several other minor QTLs located on chromosomes 3, 4, and 12 have a strong associations with aroma reported [11]. In a similar manner, comparative aroma profiling in rice identified novel aromatic compounds like alkanals, alk-2-enals, alka (E)-2, 4-dienals, 2-pentylfuran, 2-acetyl-1-pyrroline, and 2-phenylethanol.

India has a huge asset of diferent aromatic rice in both Basmati (Group V) and *indica* gene pools. There are regional specific aromatic rice, namely, Basmati (UP, Punjab, Bihar, and Haryana), Kalanamak (Eastern UP), Seeraga samba (Tamil Nadu), Jeerasala/Ganda sala (Kerala), and Chakhao Amubi/Chakhao Poireiton (North East India). Genomic analysis of Seeraga samba identified a novel mutation in OsBADH2 leading to aroma [14]. Sensory evaluation of a few of the above aromatic rice grains revealed the presence of a distinct aroma when compared to 2AP possessing Basmati (unpublished data). When compared to measuring the allelic diversity of OsBADH2, only a few attempts have been made in profiling aromatic compounds with fragrance traits in rice. Identification of novel aromatic compounds contributing to fragrance in rice and subsequent genetic analysis will accelerate the development of high-yielding fragrant rice varieties for the export market. In this study, attempts were made to profile the aromatic volatile compounds in three contrasting rice genotypes, namely, Improved White Ponni (nonaromatic fine grain variety), Pusa Basmati (aromatic long slender rice), and Chakhao Amubi (aromatic black rice from North East India).

The article "Untargeted Metabolite Profiling of Specialty Rice Grains Using Gas Chromatography Mass Spectrometry" was published in 2022. Journal: Int J Anal Chem.

## 2. Materials and Methods

### 2.1. Genetic Materials Used

Three different rice genotypes, namely, Improved White Ponni (nonaromatic indica*),* Chakhao Amubi (aromatic black rice of North East India), and Pusa Basmati 1 (aromatic long slender basmati) were used in this study. Sensory evaluation test was used as reported by Hien et al. (2006) 1.7 percent potassium hydroxide (KOH) for analyzing scent from grains of Chakhao Amubi and Pusa Basmati 1. One gram of dehusked seeds was powdered using a mortar and pestle. The samples were transferred to petri dishes containing 10 mL of 1.7% potassium hydroxide solution. The petri dishes were closed and retained at room temperature for 10 min. After 10 minutes, the dishes were opened and smelled. The presence or absence of aroma was scored (Hien et al., 2006). A sensory evaluation tests in the grains of the above 3 rice genotypes revealed that the aroma in the grains of Chakhao Amubi differed strikingly from Pusa Basmati 1 (unpublished data).

### 2.2. Profiling Volatiles in the Grains of Contrasting Rice Genotypes through GC-MS

#### 2.2.1. Sample Preparation and Volatile Capturing

Freshly harvested, dehusked grains of Chakhao Amubi, Pusa Basmati 1, and Improved White Ponni was used. 10 g dehusked seeds were ground into powder using a clean blender. Fine rice flour was transferred to a sterile conical flask containing 100 ml of 1.7% potassium hydroxide. The conical flask was tightly closed with a rubber cap containing a collector tube and sealed with a parafilm wrap to avoid any leakage. For extraction and collection of volatiles, the powered rice of three genotypes was exposed separately using 1.7% potassium hydroxide, and released volatiles were captured using stainless steel ATD prepackaged sample collection tubes containing Sorbent: Tenax GR. The conical flask containing the sample was kept at room temperature (27–30°C) overnight (8 hours) to facilitate the collection of the volatiles in the collector tube. Sorbent tubes containing trapped volatiles were removed from the flask and directly fed into the GC-MS.

The article "Untargeted Metabolite Profiling of Specialty Rice Grains Using Gas Chromatography Mass Spectrometry" was published in 2022. Journal: Int J Anal Chem.

### 2.3. GC–MS Analysis

Gas Chromatography-Mass Spectrometry (GC-MS) was performed using a Clarus SQ 8C GC/Mass Spectrometer (Perkin Elmer, USA). Nonpolar, standard, DB-5  ms capillary columns with a dimension of 30  Mts *X* 0.25 um were used. Helium (He) gas was used as a carrier. The temperature program was set at 75° C and ramped to 260° C at 10°C/min, with a hold for 2  min. The source and transfer temperatures were set to 220°C and 250°C, respectively. Identification of compounds was performed by data acquisition and evaluation using the PerkinElemer Turbo Mass software Ver6.1.0. The GC-MS analysis was obtained by matching the retention time of mass spectra and compared with the reference mass spectra in the NIST library database.

## 3. Results and Discussion

Rice is a major staple food for more than 50% of the human population and its preference is determined by grain size, cooking quality, and aroma. Next to its grain size and cooking quality, aroma or fragrance in rice grains is a key trait determining consumer preference and market price. Several experiments have concluded that aroma in rice is determined by 1-(3, 4-dihydro-2H-pyrrol-5-yl) ethanone commonly known as 2-acetyl-1-pyrroline (2AP) [9, 15]. Production and accumulation of 2AP in rice are attributed to loss-of-function mutations in the coding region of the fragrance gene, namely, OsBADH2 (Os08g0424500) [12, 16]. Any interference in the expression of OsBADH2 in nonaromatic rice led to an accumulation of 2AP and thereby enhanced aroma [17, 18] and it is overexpression reduced the level of aroma [19]. Independent genetic studies have identified multiple alleles that have been found in the same FGR gene in different genetic backgrounds and the level of aroma differs between varieties.

India is a home for scented rice varieties, and ancient records documented the cultivation of more than 300 aromatic rice varieties in various states of India [20]. Some of the regional specific aromatic rice's include Basmati (North West India), Kalanamak (Uttar Pradesh), Dubraj and Chinnor (Madhya Pradesh), Ambemohor (Maharastra), Radhunipagla (West Bengal), Jeeragasamba (Tamil Nadu), Gandhakasala (Kerala), Kalajira (Odisha), and Chakhao Amubi and Chakhao angouba (Manipur). Scented rice varieties of India differ greatly in their grain size and aroma. The majority of the scented rice is thermo/photo sensitive and short-grained and a few of them or long-grained. Aromatic and nonaromatic rice were classified mainly based on the content of 2 AP. Studies at IIRR, Hyderabad identified a few aromatic rice genotypes like Tarenbogh, Bansphool, Adamchini, and Ganjeikalli with no deletion in OsBADH2 and possessing no 2AP [21]. Ancient literature described five distinct types of scented rice, including mahasali, sugandhika, promodhaka, and pundrika. Grouping of aromatic rice genotypes based on isozyme banding pattern detected six different groups of scented rice [22], Similarly, previous studies have reported varying types of gene actions including monogenic, digenic, and trigenic interactions controlling aroma in rice. This indicated the existence of allelic, genic, and metabolomic diversity underlying fragrance in rice.

The article "Untargeted Metabolite Profiling of Specialty Rice Grains Using Gas Chromatography Mass Spectrometry" was published in 2022. Journal: Int J Anal Chem.

Profiling volatiles and semi-volatiles in aromatic rice grains detected more than 500 compounds [23]. GC-MS and LC-MS tools are becoming powerful means of profiling volatiles and metabolites. Recent advancements in sampling, collection of volatiles, and mass spectrometry identification have detected several flavor components in rice [24]. More than 40 compounds based on their mass spectra and temperature-programmed retention indices have been identified. Since 1983, 2-acetyl-1pyrroline has been regarded as the solely most important compound responsible for the aroma of rice [4]. But, a few of the aromatic rice varieties, namely, Kao Dok MAli 105/Thai Jasmine rice and Mentik Wangi, were found to possess other aromatic compounds, namely, hexanal and 2-pentylfuran.

Phylogenetic analysis using isozyme profiles revealed that aromatic rice belongs to a distinct (Group V) cluster [22, 25]. The most popular aromatic rice includes Basmati rice from India/Pakistan, jasmine rice from Thailand, and Sadri rice from Iran. Apart from this, as discussed earlier, a few of the regional specific cultivars of India have a distinct aroma and metabolic signatures. North-Eastern India harbors greater diversity of >10,000 diverse rice cultivars including both aromatic and nonaromatic rice [26, 27]. Among them, the Chakhao cultivars of Manipur are known for their pleasant aroma and several medicinal values [28]. Few studies have attempted to analyze the metabolite diversity of different Chakhao rice types in North East India [29, 30] but no studies have attempted to profile their aroma.

Our preliminary studies through sensory evaluation tests revealed the presence of a distinctive aroma/flavor in Chakhao Amubi in comparison with other aromatic rice varieties, including Basmati. This study was aimed at profiling volatile fractions of Chakhao Amubi along with Basmati (Pusa Basmati 1) and nonaromatic rice Improved White Ponni using thermal desorption gas chromatography-mass spectrometry.

### 3.1. Volatiles of Rice Grains Differing in Their Aroma

GC-MS analysis of aromatic and nonaromatic rice genotypes identified more than 50 volatile compounds (Figure 1; Table 1). Out of these 50 compounds, about 10 compounds including Hexanal, o-Xylene, 2-pentylfuran, Nonanal, Undecane, 4, 7-dimethyl-cedrene, and Dodecane, were found in all three rice genotypes (Table 1). 2-pentylfuran is found to have a nutty bean odour and is also found in various food substances like alcoholic beverages, coffee, potatoes, tomatoes, and soybean oil. It imparts a floral, fruity, nutty, and caramel-like aroma to rice [31]. 2-pentylfuran was reported as the key volatile compound in jasmine rice and Mentik Wangi [42]. In many food additives, 2-pentylfuran is used as an aromatic agent. Benzaldehyde also provides a sweet, nutty flavor [31]. Hexanal is reported to be formed from the degradation of lipid products [31] and reported to emit a green grassy odour and is associated with off-flavor in rice [4]. Dimethyl trisulfide emits a sulfury, cabbage-like odour.

The article "Untargeted Metabolite Profiling of Specialty Rice Grains Using Gas Chromatography Mass Spectrometry" was published in 2022. Journal: Int J Anal Chem.

### 3.2. Pusa Basmati and Chakhao Amubi Differ in Their Aroma Profile

There were around 30 volatile compounds specific to the aromatic genotypes Pusa Basmati 1 and Chakhao Amubi (Table 1). Among them, 11 volatiles including 2AP were found to be specifically present in Pusa Basmati 1 (Table 1). Volatiles, namely, Nonane, 1-Pentanol, octanoic acid, 2-methyl-Dimethyl trisulfide, Benzaldehyde, 2-hydroxy-acetic acid, octyl ester Dodecane, Isolongifolene-5-ol, pentadecane, pentanal, and 2 Acetyle-1 pyrroline were found to be specifically present in the grains of Pusa Basmati. These results clearly indicated the presence of 2AP (C6H9NO), a potent aromatic compound along with other volatiles present only in aromatic Pusa Basmati 1 and not observed in Chakhao Amubi and Improved White Ponni. Several researchers have previously reported 2-acetyl-1-pyrroline as the main aromatic compound in rice [15, 31, 44], P. *Amaryllifolius* [47], sorghum [44], vegetable soybean [48], and cereal coffee brew [49].

Grains of a nonbasmati rice Chakhao Amubi native of North East India were found to possess several volatiles, namely, Toluene, p-Xylene, 1,2-Dimethylbenzene, Mesitylene, Decane, Octanal, Undecane, 2-pentynal, 2-hydroxy-Benzaldehyde, Ethyl Acetate, and beta-elemene. Interestingly, the promising candidate 2AP was absent in the grains of Chakhao Amubi. Volatile compounds detected in the grains of Chakhao Amubi have been reported earlier in other aromatic rice varieties[32–35, 50].

### 3.3. Chakhao Amubi Possess Novel Aromatic and Therapeutic Compounds

Generally, black rice is believed to be rich in nutraceutical compounds and hence, they were considered medicinal rice. Manipuri Chakhao rice genotypes have been assigned geographical indication (GI) status by the Government of India (GoI, 2019). Very few studies have been carried out to document the antioxidant, anthocyanin, phenolic compounds, and few other secondary metabolites of Chakhao rice genotypes [29, 30, 51]. In this study, GC-MS analysis of the grains of Chakhao Amubi identified novel therapeutic compounds, namely, Mesitylene and *β*-elemene which are not present in the other aromatic (Pusa Basmati 1) and nonaromatic (Improved White Ponni). Mesitylene is a colorless liquid with a sweet aromatic odor. It is found to be present in several plants, including white tea [19].

The article "Untargeted Metabolite Profiling of Specialty Rice Grains Using Gas Chromatography Mass Spectrometry" was published in 2022. Journal: Int J Anal Chem.

Elemenes are natural chemical compounds found in a wide variety of plants [52]. The elemenes, consisting of *α*-, *β*-, *γ*-, and *δ*-elemene, are structural isomers and contribute to the aromas of some plants and are used as pheromones by some insects. *β*-elemene is a primary component of *Curcuma wenyujin,* exhibiting antitumor activity [53]. *β*-elemene is transformed from its precursor germacrene A, which is synthesized by germacrene A synthase (GAS). Our study has identified the biosynthesis of *β*-elemene from a cereal crop for the first time. Further studies are required to unravel the bio-synthetic pathway leading to the accumulation of *β*-elemene Chakhao Amubi, which will in turn the pave way for introducing this novel trait into other popular rice varieties through marker-assisted breeding and metabolic engineering.

## 4. Conclusion

The present study revealed key differences in the volatile profile between different aromatic and nonaromatic rice varieties. This study has documented more than fifty volatile compounds in three different rice varieties differing in their aroma (Table 1). As reported earlier, 2AP was found to be the principal volatile responsible for the fragrance in Pusa Basmati 1. The delicacy of North East India, Chakhao Amubi was found to contain novel aromatic compounds, namely, pentanal, hexanal, 2-pentylfuran, pyridine, (Z)-7-Decenal, Mesitylene, and *β*-elemene which may be responsible for its distinct flavor and therapeutic clues. Overall, this study has identified a rice genotype, Chakhao Amubi, having the ability to accumulate or synthesize novel aromatic compounds, which will enable the molecular geneticist to understand the genetic and molecular basis of these useful properties. Above all, this study has detected Chankhao Amubi possessing a potential therapeutic compound *β*-elemene which needs further investigation. The present study identified valuable volatile aromatic compounds in the grains of Chakhao Amubi, which require further quantification. Identification of genes and pathways involved in the synthesis of these volatiles can be further investigated.

The article "Untargeted Metabolite Profiling of Specialty Rice Grains Using Gas Chromatography Mass Spectrometry" was published in 2022. Journal: Int J Anal Chem.

## Figures and Tables

**Figure 1:** Chromatographs of (a) Chakhao Amubi (b) Improved White Ponni, and (c) Pusa Basmati 1.

**Table 1:** List of volatile compounds identified in grains of Chakhao Amubi, Improved White Ponni, and Pusa Basmati 1 cultivars.

Group	Volatile aromatic compound	Reference
Compounds detected in the grains of all the three genotypes (Chakhao Amubi, Pusa Basmati 1, and Improved White Ponni)	Hexanal, o-Xylene, 2-pentylfuran, nonanal, undecane, 4,7-dimethyl-cedrene, and dodecane	[31–39]
Compounds detected in the grains of Pusa Basmati 1 alone	Nonane; 1-pentanol; octanoic acid; 2-methyl-, dimethyl trisulfide; benzaldehyde; 2-hydroxy-, acetic acid; octyl ester dodecane; isolongifolene-5-ol; pentadecane; pentanal, and 2 acetyle-1 pyrroline (2AP)	[31, 32, 34–41]
Compounds detected in the grains of Chakhao Amubi alone	Toluene; p-xylene; 1,2-Dimethylbenzene; mesitylene; decane; octanal; undecane; 2-pentynal; 2-hydroxy-benzaldehyde Ethyl acetate; and beta-elemene	[23, 31, 32, 34–39, 42, 43]
Compounds common to both Chakhao Amubi and Pusa Basmati	Benzaldehyde; (Z)-7-decenal; and tetradecane	[34, 35, 37–40, 42, 44]
Compounds identified in Chakhao Amubi and Improved White Ponni	2-Methylfuran; m-xylene; decanal; pentadecane	[31, 34, 36–40, 43, 45]
Compounds identified in Pusa Basmati and Improved White Ponni	Benzothiazole	[32, 37, 39, 46]

## Data Availability

No data were used to support this study.
